The article "Application of Ultrasound Combined with Magnetic Resonance Imaging in the Diagnosis and Grading of Patients with Prenatal Placenta Accreta" was retracted in 2023. Reasons: unreliable results or conclusions; lack of ethics approval or compliance; concerns about the data; concerns about the peer review.

# Application of Ultrasound Combined with Magnetic Resonance Imaging in the Diagnosis and Grading of Patients with Prenatal Placenta Accreta

**DOI:** 10.1155/2022/1199210

**Published:** 2022-07-22

**Authors:** Xiaoyan Zhang, Fengfeng Liu, Xiaoyan Wang

**Affiliations:** Department of Obstetrics and Gynecology Women and Children's Hospital of Chongqing Medical University, China

## Abstract

In order to study the clinical application value of placenta accreta (PIA) diagnosis and grading, the authors propose a method based on ultrasound combined with magnetic resonance imaging in the diagnosis and grading of prenatal placenta accreta patients. This method is adopted in materials and methods: a retrospective analysis of hospital patients with high suspicion of placenta accreta by clinical or ultrasonography between October 2019 and October 2021, the imaging and clinical data of 312 patients who underwent placental MRI examination. The MRI imaging data of all patients were jointly analyzed, and the main observation indicators are as follows: (1) dark zone in the placenta, (2) disruption of the border of the myometrium, (3) disruption of the myometrium, (4) abnormal blood vessels in the placenta, (5) enlargement of the lower part of the uterus, and (6) local bulge of the bladder/or invasion of the adjacent tissues of the uterus. The results show the following: in MRI combined with ultrasonography (*P* < 0.05), there was no statistical significance in the specificity and accuracy of MRI combined with ultrasound to diagnose PIA (*P* > 0.05). The comparison of graded diagnostic accuracy showed that in ultrasound alone < MRI alone < MRI combined with ultrasound, the differences were statistically significant (*P* < 0.05). Ultrasound combined with MRI in the diagnosis of placenta accreta is in good agreement with the clinical and surgical pathological results; MRI examination can be used as an important method for prenatal placenta accreta screening. MRI can classify placenta accreta to some extent.

## 1. Introduction

Placenta accreta (PIA) is due to uterine hypoplasia or injury(Figure 1), resulting in partial loss of decidua basalis, and placental chorionic trophoblasts invade the myometrium through the missing part and even break through the serosa, involving parametrial tissues and organs, an abnormal placental implantation. Depending on the depth of implantation of the placental villi into the myometrium, divide it into three types: (1) placenta accreta (placenta accreta) refers to the placental villi attached or adhered to the superficial muscle layer, but does not invade the deep muscle layer, (2) placenta accreta (placenta accreta) refers to the implantation of the placenta into the deep muscle layer and does not reach the serosa layer, and (3) placenta accreta (placenta percreta) is when placental villi penetrate the muscularis layer and involve the serosal layer; it even involves adjacent tissues and organs, which is the most serious type [1]. Risk factors for placenta accreta are often related to endometrial trauma and endometrial dysplasia. A previous history of cesarean section (LUSC), placenta previa (PP), history of multiple miscarriages or multiple hysterectomy, and previous history of other uterine surgery are the main risk factors for placenta accreta; among them, placenta previa and the history of previous cesarean section are the most important; if the two exist together, the incidence of placenta accreta will be significantly increased. Therefore, some scholars believe that caesarean section is the most important risk factor for PIA, and the risk of placenta accreta increases with the increase in the number of caesarean sections. Because the cause of placenta accreta may be endometrial damage, in addition to cesarean section, the history of repeated uterine removal, other intrauterine surgical operations, and intrauterine infection are also risk factors for placenta accreta. Another scholar's research has shown that advanced pregnancy (age>35 years) is also one of the independent risk factors for placenta accreta. Some scholars have shown that assisted reproductive technology is another independent risk factor for placenta accreta [2].

The article "Application of Ultrasound Combined with Magnetic Resonance Imaging in the Diagnosis and Grading of Patients with Prenatal Placenta Accreta" was retracted in 2023. Reasons: unreliable results or conclusions; lack of ethics approval or compliance; concerns about the data; concerns about the peer review.

The clinical importance of PIA arises from increased maternal morbidity and mortality and massive postpartum and sometimes intrapartum or antepartum hemorrhage. When there is placenta accreta, it is difficult to separate the placenta from the uterus, sometimes requiring instrumental forceps, which can lead to massive bleeding before, during and after the operation, and the bleeding is difficult to control and can cause shock in severe cases; it can also be complicated by disseminated intravascular coagulation (DIC), uterine perforation, and subsequent severe intrauterine infection, which increases the probability of hysterectomy and even endangers the lives of mothers and babies. In recent years, the incidence of placenta accreta has increased significantly, reaching 1/533, which is 20 times higher than before. It has become an important cause of postpartum hemorrhage, perinatal emergency hysterectomy, and maternal death. According to a WHO survey on caesarean section rates in 2007-2008, among the nine Asian countries surveyed, China has the highest rate of caesarean section at 46.2%. With changes in social concepts and population policy adjustments, the age of childbearing has been delayed, and the number of “second children” has increased; many people with “second children” are advanced mothers, which may increase the incidence of placenta accreta and clinical issues that must be faced by an obstetrician [3]. Accurate prenatal diagnosis, planned cesarean section, and hysterectomy can reduce complications and mortality in pregnancy with placenta accreta. Magnetic resonance imaging (MRI), on the other hand, with its higher soft tissue resolution, comprehensive imaging information is provided before birth. Based on this, the authors intend to explore the diagnostic efficacy of MRI combined with ultrasound (US) in the diagnosis and grading of PIA, the results are reported as follows.

The article "Application of Ultrasound Combined with Magnetic Resonance Imaging in the Diagnosis and Grading of Patients with Prenatal Placenta Accreta" was retracted in 2023. Reasons: unreliable results or conclusions; lack of ethics approval or compliance; concerns about the data; concerns about the peer review.

## 2. Literature Review

Jiao and others believed that clinical symptoms, signs, and laboratory examinations of placenta accreta were of limited value, and imaging examinations became an important auxiliary diagnosis. Currently, the first-line test for obstetricians to screen for and diagnose antenatal placenta accreta is transabdominal or transvaginal color Doppler ultrasonography [4]. Ha et al., in a systematic evaluation of the value of ultrasound in the diagnosis of prenatal placenta accreta, concluded that the sensitivity of ultrasonography in the diagnosis of prenatal placenta accreta was 77%-88% and the specificity was 93%-96% [5]. Zhang et al. believe that the biggest advantage of ultrasonography is the convenience of examination, the blood flow signals of the placenta and uterus can be observed, but ultrasound also has shortcomings; for example, the soft tissue resolution and spatial resolution are relatively low, and the field of view (FOV) is small; in addition, the imaging quality of pregnant women is poor, such as obesity, oligohydramnios, and more intestinal gas in the imaging area, and the placenta is located in the posterior wall of the uterus; these factors will affect the image quality and diagnostic results to varying degrees [6]. Mcdannold et al. believe that MRI has high soft tissue resolution, no ionizing radiation, can scan in any orientation, and has a large scanning field of view, and it is not interfered by factors such as the body shape of the pregnant woman, intestinal gas, and placenta position; in the past, conventional spin echo sequence scanning was used for magnetic resonance imaging, which took a long time, and it was difficult to overcome the respiratory motion artifacts and fetal movement artifacts, which limited the application of MRI in obstetrics [7]. In the past ten years, with the development of MRI hardware and software and the application of fast scanning technology, the impact of physiological motion artifacts on image quality has been reduced, and its application advantages in prenatal examinations have become prominent, when the diagnosis of placenta accreta is not clear by ultrasonography, especially when evaluating the depth of placenta accreta and the infiltration of parametrial tissues and organs, MRI can be used as a supplementary imaging method [8]. US is the preferred auxiliary examination for obstetricians, and it is recognized as a relatively safe and effective imaging examination. For the application of MRI in prenatal examination, most researchers generally believe that it is relatively safe. However, considering the special physiological characteristics of fetal development, the embryonic development has not been completed in the first 3 months of pregnancy and is easily affected by various physical factors [9]. The SAR value of fetal magnetic resonance examination should be lower than 3 W/kg, SAR value is proportional to the square of the static magnetic field strength, 1.5T magnetic resonance SAR value is significantly lower than 3.0 T magnetic resonance, and therefore, 1.5T magnetic resonance imaging is often used in prenatal examinations. Since the body heat production caused by radio frequency pulse is mainly located on the surface of the body and is weakest in the center of the body and the amniotic fluid has a certain protective effect on the fetus, there has been no report on fetal injury [10].

The article "Application of Ultrasound Combined with Magnetic Resonance Imaging in the Diagnosis and Grading of Patients with Prenatal Placenta Accreta" was retracted in 2023. Reasons: unreliable results or conclusions; lack of ethics approval or compliance; concerns about the data; concerns about the peer review.

## 3. Methods

### 3.1. Analysis Objects

From October 2019 to October 2021, 312 pregnant women who gave birth in our hospital and were diagnosed with placenta accreta by intraoperative clinical diagnosis and postoperative pathological diagnosis were selected as the research objects, the age ranged from 22 to 38 years, with an average of 26.98 ± 5.85 years old, the gestational age was 30 to 38 weeks, with an average of 35.69 ± 2.58 weeks, and the pregnancy was 1 to 5 times, with an average of 2.69 ± 2.69 ± 2.58 weeks. The parity was 1 to 4 times, with an average of 2.08 ± 0.87 times, 280 cases had a history of cesarean section, 20 cases had a history of myomectomy, and 12 cases had a history of other uterine cavity operations; all pregnant women were clearly conscious, without serious cardiovascular and cerebrovascular diseases, abnormal liver and kidney functions, coagulation disorders, and mental disorders [11].

### 3.2. Analysis Method

#### 3.2.1. US Examination and Graded Diagnosis

Using Philips iU22 color US diagnostic system, with a probe frequency of 3.5 Hz, two US professional deputy chief physicians performed US images to assess whether there was placenta accreta, and the cases diagnosed with placenta accreta were classified according to the previous literature: In Grade I, the retroplacental space disappears and is occupied by placental tissue, the strong echo lines of the decidua disappear, and the myometrium becomes thin (<2 mm). In Grade II, in addition to the manifestations of Grade I, the myometrium disappears, and there are venous pools of different sizes in the placenta, which are the same as the abnormally dilated blood vessels on the uterine wall after the placenta [12]. In Grade III, in addition to grade II manifestations, the uterine serosa layer is interrupted, local blood vessels and solid mass shadows protrude to the bladder, the posterior wall of the bladder is not smooth or uneven, and at the same time, the authors classified cases where US failed to diagnose placenta accreta as Grade 0. If the evaluations are consistent, the consistency evaluation results will be accepted [13]. If there are differences in the evaluation results, the two evaluating physicians will reach a consensus after consultation as the evaluation result.

The article "Application of Ultrasound Combined with Magnetic Resonance Imaging in the Diagnosis and Grading of Patients with Prenatal Placenta Accreta" was retracted in 2023. Reasons: unreliable results or conclusions; lack of ethics approval or compliance; concerns about the data; concerns about the peer review.

#### 3.2.2. MRI Examination and Graded Diagnosis

Philips Achieva 1.5t dual gradient superconducting magnetic resonance equipment (maximum gradient field intensity 66 mm/Tm, maximum gradient switching rate 180 T/m/s, and climbing time 0.18 ms, AchievaNovalDual) and 16-channel body phase controlled front ring were adopted. T1-weighted imaging (T1WI) was performed using a gradient echo sequence [repetition time (TR): 500 ms, echo time (TE): 14 ms]. T2-weighted imaging (T2WI) was performed using a single excited fast spin echo sequence (TR: 1800 ms, TE:12 ms) and a short reversal time reversal recovery (STIR) sequence (TR: 1600 ms, TE: 70 ms) [14]. Imaging parameters are as follows: matrix of 256 × 256, acquisition times of 2~3 times, slice thickness of 3~5 mm, and slice spacing of 0.5~1.0 mm. The pregnant woman is in a supine position, her feet are advanced, and her bladder is moderately full; combined with the previous literature, the coronal orientation of the pelvic cavity of pregnant women is upward, and the pelvic sagittal, coronal, and axial scans are performed. 312 cases underwent contrast-enhanced scanning, magnetic resonance contrast agent (Gd-DTPA), dose 0.1 mmol/kg, injected through cubital vein, firstly underwent T1WI cross-sectional dynamic enhanced scanning, and then underwent sagittal and coronal scanning. The scan parameters are the same as the TIWI scan sequence above [15], the scanning range is from about 2 cm above the uterine fundus to the pubic symphysis. Diagnosis was made by two senior radiologists who were unaware of surgical and pathological results, and the placenta morphology, location, signal intensity, implantation site, uterine wall, and adjacent organs were observed in MRI. Combined with a previous literature, placenta accreta was divided into three grades according to MRI findings: in Grade I: MRI sees that the placenta is still in a regular shape, clearly demarcated with the uterine wall, and the bladder wall is smooth. In Grade II, MRI shows abnormal placenta signal, low signal in the placenta on T2WI, the placenta implantation is located in the uterine wall, and the bladder wall is smooth [16]. In Dish grade, MRI shows placenta accreta, and the placenta implantation invades the pelvic organs, such as the bladder. Invasion, local nodular changes in the bladder wall. At the same time, the authors classified cases where MRI failed to diagnose placenta accreta as grade 0.

The article "Application of Ultrasound Combined with Magnetic Resonance Imaging in the Diagnosis and Grading of Patients with Prenatal Placenta Accreta" was retracted in 2023. Reasons: unreliable results or conclusions; lack of ethics approval or compliance; concerns about the data; concerns about the peer review.

#### 3.2.3. MRI Combined with US Diagnosis and Grading Diagnosis

Prenatal MRI was combined with US diagnostic grading results, determined by discussion and consultation between 1 radiologist and 1 US physician. If the diagnostic grades of the two physicians are the same, this grade is used as the combined diagnostic grade; if the US and MRI physicians have different diagnostic grades [17], the US shall prevail for Grades 0 and I, and the MRI grades shall prevail for Grades II and III.

#### 3.2.4. Pathological Examination

First, the tissue was grossly observed, then HE stained smears and microscopic observation. Histopathologically, it is confirmed whether there is placenta accreta [18]. If there is, according to the degree of placental villi invading the myometrium, it is divided into 3 types: adhesion, accreta, and penetrating placenta. At the same time, they were, respectively, defined as follows: placenta accreta was Grade I, placenta accreta was Grade II, and placenta penetratus was Grade III.

#### 3.2.5. Image Processing and Evaluation Criteria

Under the condition of not knowing the results of pathological examination, the single-blind method was used to read the films, and the MRI images focused on analyzing the signal in the placenta, the relationship between the placenta and the myometrium, the localized swelling or thinning of the uterus, the swelling of the lower segment of the uterus, the relationship between the placenta and the cervix [19], and the tortuosity in the placenta, dilated vascular shadow, comprehensive consideration, and interpretation. The diagnosis of PIA is based on the Masselli pathological classification: (1) adhesion—the placental villi are attached to the myometrium without infiltration; (2) implantation—the placental villi invade the myometrium without reaching the serosa; and penetrating—the placental villi went through the muscularis to reach or penetrate the serosa.

The article "Application of Ultrasound Combined with Magnetic Resonance Imaging in the Diagnosis and Grading of Patients with Prenatal Placenta Accreta" was retracted in 2023. Reasons: unreliable results or conclusions; lack of ethics approval or compliance; concerns about the data; concerns about the peer review.

### 3.3. Statistical Analysis

Statistical method SPSS16.0 software was used for statistical analysis of the data, and the measurement data was represented by xts; Prenatal MRI, US diagnosis and MRI combined with US diagnosis were performed by chi-square test, respectively [20]; The Kappa test was used to test the consistency of prenatal USMRI diagnostic grading, MRI combined with US diagnosis and postoperative pathological grading, and the Kappa coefficient was used to test the consistency of the two evaluation results, good agreement, Kappa ≥0.7 indicates strong agreement.

### 3.4. Analysis of Results

There was no statistical significance in the comparison of the sensitivity of the three examination schemes for diagnosing PIA, however, the specificity and accuracy of ultrasound alone in diagnosing PIA were significantly lower than those of MRI alone, MRI combined with ultrasound examination, and the differences were statistically significant (P <0.05), there was no statistical significance in the specificity and accuracy of MRI combined with ultrasound to diagnose PIA (P >0.05), as shown in Table 1.

The comparison of the grading diagnostic accuracy showed that the difference was statistically significant between ultrasound alone < MRI alone < MRI combined with ultrasound (*P* < 0.05), as shown in Table 2.

As can be seen from Table 3, among the 312 patients with placenta accreta, 187 were diagnosed with placenta accreta by prenatal MRI combined with US [21], with a diagnostic rate of 86.27%, which was higher than the diagnostic coincidence rate of placenta accreta by prenatal MRI alone (76.47%), and the difference was statistically significant (*X*^2^ = 53.536, *P* = 0.00). The degree of agreement between the combined diagnostic grading and postoperative pathological grading was strong (kappa = 0.842, *P* = 0.000).

After comparing the gold standard data of surgical or pathological diagnosis, it was found that the index of magnetic resonance imaging in the diagnosis of placenta accreta was 74%, which was slightly higher than that of color Doppler diagnostic index of 60.5%; there was no significant difference in the diagnostic index between the two groups (*P* > 0.05) [22]. The kappa value of magnetic resonance imaging was 0.739, and the kappa value of acoustic Doppler was 0.610, both > 0.4, which were consistent with the gold standard, as shown in Table 4.

Ultrasound features with high sensitivity and specificity are as follows: placental lacuna and partial or complete disappearance of the retroplacental space, with a sensitivity of 92.1% and 79.4% and a specificity of 73.9% and 65.2%, respectively. The features with high sensitivity and specificity in MRI were irregular enlargement and deformation of uterine volume; the sensitivity and specificity were 87.3% and 87.0%; the second was the thinning or disappearance of the dark zone in the placenta and the myometrium on T2-weighted images; the sensitivity and specificity were 79.4%, 79.4%, and 69.6%, 78.3%, respectively. See Figure 2.

The article "Application of Ultrasound Combined with Magnetic Resonance Imaging in the Diagnosis and Grading of Patients with Prenatal Placenta Accreta" was retracted in 2023. Reasons: unreliable results or conclusions; lack of ethics approval or compliance; concerns about the data; concerns about the peer review.

## 4. Discussion

Placenta accreta refers to the invasion of placental villi into the myometrium due to primary decidual hypoplasia or traumatic endometrial defect, which can lead to severe postpartum hemorrhage, uterine perforation, and secondary infection and is a common emergency in obstetrics [23]. Pathologically, it is divided into 3 types according to the severity of placental villi invading the muscularis: placenta accreta, placenta accreta, and placenta penetra. Different degrees of placenta accreta have completely different treatment methods. Placenta accreta and placenta penetrance are often the main culprits that lead to postpartum hemorrhage, uterine perforation, and coinfection; therefore, early, noninvasive, and accurate diagnosis and grading of placenta accreta have very important clinical guiding value.

Ultrasound is an imaging method represented by noninvasive, simple, nonradiation, and low-cost characteristics and has become an indispensable examination link during pregnancy. Relevant studies suggest that after the occurrence of PIA, the placenta can show abnormal thickening echo signs under ultrasound, and the hypoechoic zone of the myometrium at the attachment site becomes thin or even disappears, and due to the formation of venous blood pool, there are often multiple anechoes of different sizes and shapes in the placenta. In the recessed area, for pregnant women with placenta previa, the increase in gestational age was not accompanied by an upward shift in the echogenicity of the lower edge of the placenta. In this study, there was little difference in the sensitivity of the three examination schemes for the diagnosis of PIA, and the specificity and accuracy of the ultrasound examination scheme were significantly lower than those of MRI alone and MRI combined with ultrasound examination, which indicated that MRI was more suitable for the diagnosis of PAI, although the PIA placental parenchyma is usually accompanied by focal lacunar blood flow under color Doppler ultrasound, and the basal facial venous plexus is rich in signal; the acoustic signal is easily disturbed by the abdominal fat layer [24], amniotic fluid, and fetal bone, and even the position of the placenta, the beam attenuation, and absorption are significant, so the resolution of soft tissue is far inferior to that of MRI, which hinders accurate preoperative diagnosis. Relevant experts suggested that for pregnant women with suspected PIA diagnosed by ultrasound, MRI should be used as a routine examination, which can guide the rational choice of delivery mode after early diagnosis and provide direct anatomical evidence for the design of cesarean section.

The article "Application of Ultrasound Combined with Magnetic Resonance Imaging in the Diagnosis and Grading of Patients with Prenatal Placenta Accreta" was retracted in 2023. Reasons: unreliable results or conclusions; lack of ethics approval or compliance; concerns about the data; concerns about the peer review.

MRI is more expensive and takes longer to scan; it is far less widely used in prenatal examination than ultrasound, but because of its high resolution of soft tissue, large imaging range, and more flexible orientation, it has positive significance for the diagnosis of PIA and the evaluation of implantation depth. According to relevant literature reports, the T2WI sequence of MRI can fully demonstrate the thinning and interruption of the myometrium and the nodular hyperintensity sign in the hypointense myometrium, and the serrated degeneration of the interface is more common in adhesive PIA; the placenta can be peeled off with bare hands, which can cause the placental surface to be rough and associated with a lot of blood oozing. Implantable PIA can find that the myometrium and placental tissue are fused with each other, and a large resistance can be felt when peeling off with bare hands; if the peeling is unsuccessful or the bleeding is excessive, hysterectomy should be planned. Penetrating PIA shows that the uterus and bladder wall are not intact, and it is impossible to dissect the uterus by hand; it is necessary to be careful to avoid uterine rupture and properly formulate a hysterectomy operation plan. This study found that prenatal application of MRI combined with ultrasound can obtain a more prominent PIA grading diagnosis effect, suggesting that the combined diagnosis can carry out multifaceted analysis of the PIA implantation depth, and objective selection of consistent diagnostic information can more accurately reflect the actual situation. And the degree of disturbance is not strongly correlated with the depth of placenta accreta; the diagnostic efficiency of color Doppler ultrasound in grading PIA is insufficient; although MRI has higher resolution, with the increase of gestational age, the difference of T2WI signal between placental stroma and placental lobule becomes more and more prominent, resulting in uneven internal signal, which may increase some false negative cases; therefore, the combined application of multiple imaging methods is more necessary [25].

## 5. Conclusion

Prenatal MRI combined with US examination can better detect patients with placenta accreta, can reflect the basic pathological features of placenta accreta, and can better show the site of placenta accreta, the depth of invasion, and the involvement of adjacent organs. Prenatal MRI combined with US examination may play an important role in the graded diagnosis of placenta accreta, the setting of treatment plans, and the evaluation of efficacy; at the same time, it can provide an accurate imaging basis for the formulation of clinical surgical plans. In conclusion, both prenatal magnetic resonance imaging examination and ultrasonography have high diagnostic value for placenta accreta, and magnetic resonance imaging examination has a slight advantage, which can play a supplementary role in the diagnosis of placenta accreta by ultrasonography.

The article "Application of Ultrasound Combined with Magnetic Resonance Imaging in the Diagnosis and Grading of Patients with Prenatal Placenta Accreta" was retracted in 2023. Reasons: unreliable results or conclusions; lack of ethics approval or compliance; concerns about the data; concerns about the peer review.

## Figures and Tables

**Figure 1:** Placenta implantation.

**Figure 2:** Sensitivity of ultrasound- and MRI-related features.

**Table 1:** Results of MRI, ultrasound, and their combined examination to confirm the diagnosis of PIA (cases).

Check the scheme		Postpartum pathological detection			Sensitivity (%)	Specificity (%)	Accuracy (%)
		Negative	Negative	Negative			
Simple MRI	Negative	64	45	79	62.79	87.76	81.99
	Positive	43	251	283			
	Total	79	271	372			
Simple ultrasound	Negative	60	71	141	69.77	71.68	71.24
	Positive	25	205	201			
	Total	76	217	317			
The MRI was combined with the ultrasound procedure	Negative	53	26	88	72.09	90.91	86.56
	Positive	23	260	284			
	Total	76	286	372			

**Table 2:** The results of MRI, ultrasound, and their combined examinations for grading diagnosis of PIA [cases (%)].

Check the scheme		Postpartum pathological detection				Accuracy (%)
		Adhesive	Implantable	Penetrability	Total	
Simple MRI	Negative	33	9	0	33	52.16%
	Adhesive	26	5	0	23	
	Implantable	3	19	5	34	
	Penetrability	0	0	9	9	
	Total	62	33	11	86	
Simple ultrasound	Negative	32	4	0	26	35.05%
	Adhesive	8	10	1	21	
	Implantable	7	13	2	32	
	Penetrability	3	6	8	27	
	Total	52	33	21	76	
The MRI was combined with the ultrasound procedure	Negative	31	4	0	22	65.28%
	Adhesive	41	2	0	23	
	Implantable	1	32	1	38	
	Penetrability	0	1	10	11	
	Total	42	33	11	86	

**Table 3:** The graded diagnosis and pathological comparison of placenta accreta by prenatal MRI.US and combined diagnosis.

	Placental implantation grade n			
	Level 0	Level I	Level II	Level III
Pathologic diagnosis	0	21	43	20
MRI diagnose	33	34	24	16
US diagnose	20	15	35	23
MRI in combination with US diagnosis	7	15	32	9

**Table 4:** Evaluation of ultrasound and MRI in the diagnosis of placenta accreta (%).

Group	False yang rate	False yin rate	Positive predictive value	Negative predictive value
Ultrasound group	7.2	31.2	78	83.5
The US was combined with the MR group	7.8	32.2	81	90.5

## Data Availability

The data used to support the findings of this study are available from the corresponding author upon request.

The article "Application of Ultrasound Combined with Magnetic Resonance Imaging in the Diagnosis and Grading of Patients with Prenatal Placenta Accreta" was retracted in 2023. Reasons: unreliable results or conclusions; lack of ethics approval or compliance; concerns about the data; concerns about the peer review.

## References

[1] Solomon O., Cohen R., Zhang Y. (2020). Deep unfolded robust PCA with application to clutter suppression in ultrasound. *IEEE transactions on medical imaging*.

[2] Waqar H., Riaz R., Ahmed N. M., Majeed A. I., Abbas S. R. (2022). Monodisperse magnetic lecithin-pfp submicron bubbles as dual imaging contrast agents for ultrasound (us) and mri. *RSC Advances*.

[3] Raj M. H., Mullins J. N., Chi J. M., Choy A. H., Grimaldi G. M., Friedman B. (2020). The utility of abdominopelvic CT in pregnant patients with abdominal pain and a negative or inconclusive abdominal MRI. *Clinical Imaging*.

[4] Jiao J., Namburete A. I., Papageorghiou A. T., Noble J. A. (2020). Self-supervised ultrasound to MRI fetal brain image synthesis. *IEEE Transactions on Medical Imaging*.

[5] Ha I. Y., Wilms M., Handels H., Heinrich M. P. (2019). Model-based sparse-to-dense image registration for realtime respiratory motion estimation in image-guided interventions. *IEEE Transactions on Biomedical Engineering*.

[6] Zhang Y., Dong Y., Fu H., Huang H., Sun Y. (2020). Multifunctional tumor-targeted PLGA nanoparticles delivering Pt(IV)/sibirc5 for US/MRI imaging and overcoming ovarian cancer resistance. *Biomaterials*.

[7] McDannold N., White P. J., Cosgrove G. R. (2020). Using phase data from MR temperature imaging to visualize anatomy during MRI-guided focused ultrasound neurosurgery. *IEEE transactions on medical imaging*.

[8] Luijten B., Cohen R., Bruijn F., Schmeitz H., Sloun R. (2020). Adaptive ultrasound beamforming using deep learning. *IEEE Transactions on Medical Imaging*.

[9] Wang Y., Liu Y., Wu H., Zhang J., Tian Q., Yang S. (2019). Functionalized holmium-doped hollow silica nanospheres for combined sonodynamic and hypoxia-activated therapy. *Advanced Functional Materials*.

[10] Bekoulis T., Apostolopoulos A. P., Papatheodorou A., Lakiotaki E., Papanikolaou A. (2021). Primary extranodal skeletal-muscle non-Hodgkin b cell lymphoma: clinical presentation and diagnostic approach. *Journal of Long-Term Effects of Medical Implants*.

[11] Dong Q., Wan C., Yang H. (2020). Targeted gold nanoshelled hybrid nanocapsules encapsulating doxorubicin for bimodal imaging and near-infrared triggered synergistic therapy of Her2-positve breast cancer. *Journal of Biomaterials Applications*.

[12] Stember J. N., Terilli K. L., Perez E. (2020). Surface point cloud ultrasound with transcranial Doppler: coregistration of surface point cloud ultrasound with magnetic resonance angiography for improved reproducibility, visualization, and navigation in transcranial doppler ultrasound. *Journal of Digital Imaging*.

[13] Wang P., Du T., Wang L., Kong L., Shi Y. (2020). A low-complexity minimum variance algorithm combined with power method for ultrasound imaging. *Acoustical Physics*.

The article "Application of Ultrasound Combined with Magnetic Resonance Imaging in the Diagnosis and Grading of Patients with Prenatal Placenta Accreta" was retracted in 2023. Reasons: unreliable results or conclusions; lack of ethics approval or compliance; concerns about the data; concerns about the peer review.

[14] Li H., Porée J., Chayer B., Cardinal M. H. R., Cloutier G. (2020). Parameterized strain estimation for vascular ultrasound elastography with sparse representation. *IEEE Transactions on Medical Imaging*.

[15] Moore M. J., Sebastian J. A., Kolios M. C. (2019). Determination of cell nucleus-to-cytoplasmic ratio using imaging flow cytometry and a combined ultrasound and photoacoustic technique: a comparison study. *Journal of Biomedical Optics*.

[16] Xu X., Li L., Sharma A. (2021). Controlling messy errors in virtual reconstruction of random sports image capture points for complex systems. *International Journal of Systems Assurance Engineering and Management*.

[17] Rajendran A., Balakrishnan N., Ajay P. (2022). Deep embedded median clustering for routing misbehaviour and attacks detection in ad-hoc networks. *Ad Hoc Networks*.

[18] Liu X., Liu J., Chen J., Zhong F. (2022). Catalytic conversion and DFT analysis of post DDBD-catalysis system for degradation of toluene, ethyl acetate and acetone with different metal-oxides catalysts. *Journal of Rare Earths*.

[19] Huang R., Yan P., Yang X. (2021). Knowledge map visualization of technology hotspots and development trends in China’s textile manufacturing industry. *IET Collaborative Intelligent Manufacturing*.

[20] Zhang X., Rane K., Kakaravada I., Shabaz M. (2021). Research on vibration monitoring and fault diagnosis of rotating machinery based on internet of things technology. *Nonlinear Engineering*.

[21] di Pasquo E., Ghi T., Calì G. (2019). OP19. 09: Intracervical lakes as a sonographic marker of placenta accreta spectrum (PAS) in patients with placenta previa. *Ultrasound in Obstetrics & Gynecology*.

[22] Chiu Y. H., Lee T. S. H., Chao E. (2020). Application of classification criteria of Sjogren syndrome in patients with sicca symptoms: Real-world experience at a medical center. *Journal of the Formosan Medical Association*.

[23] Clark H. R., Ng T. W., Khan A., Happe S., Twickler D. M. (2020). Placenta accreta spectrum: correlation of mri parameters with pathologic and surgical outcomes of high-risk pregnancies. *American Journal of Roentgenology*.

[24] Xu L., Xie X., Shi X., Zhang P., Zhang B. (2021). Potential application of genomic profiling for the diagnosis and treatment of patients with sarcoma. *Oncology Letters*.

[25] Zhou K., Liu Z., He W., Cai J., Hu L. (2022). Application of 3d whole-brain texture analysis and the feature selection method based on within-class scatter in the classification and diagnosis of Alzheimer's disease. *Therapeutic Innovation & Regulatory Science*.

